# Early growth response 1 regulates glucose deprivation-induced necrosis

**DOI:** 10.3892/or.2012.2134

**Published:** 2012-11-14

**Authors:** HYUN MIN JEON, SU YEON LEE, MIN KYUNG JU, CHO HEE KIM, HYE GYEONG PARK, HO SUNG KANG

**Affiliations:** 1 Department of Molecular Biology, College of Natural Sciences, Pusan National University, Pusan 609-735, Republic of Korea; 2 Nanobiotechnology Center, Pusan National University, Pusan 609-735, Republic of Korea

**Keywords:** early growth response 1, glucose deprivation, reactive oxygen species, necrosis, multicellular tumour spheroids

## Abstract

Necrosis is commonly found in the core region of solid tumours due to metabolic stress such as hypoxia and glucose deprivation (GD) resulting from insufficient vascularization. Necrosis promotes tumour growth and development by releasing the tumour-promoting cytokine high mobility group box 1 (HMGB1); however, the molecular mechanism underlying necrotic cell death remains largely unknown. In this study, we show that early growth response 1 (Egr-1) is induced in a reactive oxygen species (ROS)-dependent manner by GD in several cell lines such as A549, MDA-MB-231 and HepG2 cells that exhibit necrosis upon GD. We found that Egr-1 short hairpin RNA (shRNA) prevented GD-induced necrosis and HMGB1 release. Necrosis-inhibiting activity of Egr-1 shRNA was also seen in multicellular tumour spheroids (MTSs), an *in vitro* tumour model system. In contrast, Egr-1 overexpression appeared to make tumour cells more susceptible to GD-induced necrosis. Finally, Egr-1 shRNA suppressed the growth of MTSs. These findings demonstrate that Egr-1 is implicated in GD-induced necrosis and tumour progression.

## Introduction

Unlike tumour suppressive apoptosis and autophagic cell death, necrosis promotes tumour growth, progression, and aggressiveness (1,2). The tumour promoting activity of necrosis is thought to be mediated by a nuclear protein high mobility group box 1 (HMGB1), which exerts pro-inflammatory and tumour-promoting cytokine activities when released into the extracellular spaces due to the rupture of the plasma membrane by necrosis (1–4). In solid tumours, the cells in the inner regions experience metabolic stress such as hypoxia and glucose deprivation (GD) resulting from insufficient vascularization. Although most cells adapt to this environment to obtain more aggressive properties, those in the core region die by necrosis, thereby forming the necrotic core (5). Because necrosis is linked to tumour growth and development, it is an important cell death type in tumour cell biology; however, the molecular mechanism underlying necrotic cell death remains largely unknown.

Early growth response 1 (Egr-1) is a 3 Cys2-His2 type COOH-terminal zinc-finger transcription factor that binds to GC-rich recognition motifs (5′-GCGT/GGGGCG-3′ or 5′-TCCT/ACCTCCTCC-3′) (6,7). Egr-1 is induced by a number of different stimuli, such as anti-cancer drugs and growth factors and inhibits or stimulates tumour growth depending the cellular context and the duration of Egr-1 induction (6–13). Egr-1 was able to directly regulate multiple tumour suppressors including p53, TGF-β1, and PTEN to induce apoptotic cell death (14). In addition, Egr-1 is induced by hypoxia and plays a critical role(s) in hypoxia-induced tumour progression, survival, and angiogenesis (15–18). Furthermore, Egr-1 is involved in hepatocyte growth factor (HGF)-induced cell scattering, migration, and invasion via Snail activation (19). While transient induction of Egr-1 is known to activate angiogenesis, sustained Egr-1 expression induces antiangiogenesis, growth arrest, and apoptosis (20). Thus, Egr-1 is thought to act as a crucial regulator of tumour cell death, growth, invasion, and angiogenesis.

In this study, we tried to identify the mechanism underlying metabolic stress-induced necrosis. Previously, we showed that GD induced necrosis in several tumour cell types including A549, MDA-MB-231, and HepG2 cells and activation of protein kinase C by treatment of phorbol 12-myristate 13-acetate (PMA) switched GD-induced necrosis to apoptosis in A549 cells (21). By cDNA microarray analysis, we found that Egr-1 expression was increased by GD, but not by GD+PMA. In this study, we evaluated the possible role(s) of Egr-1 in necrosis. We found that Egr-1 shRNA prevented necrosis, whereas Egr-1 overexpression made tumour cells more sensitive to GD, thereby leading to necrosis. In addition, Egr-1 shRNA suppressed the growth of multicellular tumour spheroids (MTSs), an *in vitro* tumour model system. Taken together, these results demonstrate that Egr-1 plays an important role(s) in GD-induced necrosis and tumour progression.

## Materials and methods

### Cell culture, chemical treatment, and multicellular tumour spheroid (MTS) culture

A549, MDA-MB-231, HepG2, HCT116, and HeLa cells were obtained from American Type Culture Collection, and maintained in RPMI-1640 or DMEM supplemented with 10% (v/v) heat-inactivated fetal bovine serum (Hyclone, Logan, UT, USA) and 1% penicillin-streptomycin (Hyclone) in a 37°C humidified incubator with 5% CO_2_. The cells were treated with GD, reactive oxygen species [ROS, including H_2_O_2_ and menadione (an O_2_^-^ generator)], or other chemicals as described previously (22). Multicellular tumour spheroid culture was performed using MCF-7 cells (provided by Dr J.I. Yook, University of Yonsei, Korea) as described previously (22) and MTSs dissociation into subpopulations of cells from four different locations was conducted as described by LaRue and colleagues (23).

### Microarray

Microarray was performed to screen the differentially expressed genes using Operon Human Whole 35K Oligo chips (GenoCheck, Korea) (22). The Affymetrix microarray data have been deposited in the Gene Expression Omnibus (GEO) database (GEO accession no. GSE24271).

### Western blotting, HMGB1 release assay, RT-PCR, and real-time PCR

Western blotting were performed using the following antibodies: Egr-1 (Santa Cruz, CA); α-tubulin (Biogenex, CA); HMGB1 (BD Pharmingen, CA); CuZnSOD (Santa Cruz, CA); ERK1/2 (Cell Signaling, MA). The HMGB1 release assay was carried out as described previously (21,22). Transcript levels were assessed with reverse transcription-polymerase chain reaction (RT-PCR) with primers for Egr-1 and GAPDH (Table I). Quantitative real-time PCR was conducted in a LightCycler (Roche Diagnostics, Mannheim, Germany) using a SYBR Green kit (Roche Diagnostics) with primers for Egr-1 and β-actin (Table I).

### Hoechst 33342 (HO)/propidium iodide (PI) staining and ROS staining

To determine the cell death mode, Hoechst 33342 (HO) and propidium iodide (PI) double staining was performed (21,22). In 2D culture, cells were seeded at a density of 2.5×10^5^ cells/ml in 35-mm dishes. After 24 h, the cells were treated with GD for the indicated times and then stained with HO (1 μg/ml) and PI (5 μg/ml) for 15 min. In 3D culture, equal numbers of spheroids were transferred to 1.2% agarose-coated 60-mm dishes and trypsinized and then stained with HO/PI, The stained cells were observed under a fluorescence microscope and apoptotic and necrotic cells were scored. Intracellular H_2_O_2_, O_2_^-^ and mitochondrial ROS measurement were conducted as described previously (21,22).

### Egr-1 transfection and short hairpin RNA (shRNA) interference

pcDNA3.1-Egr-1, constructed by inserting the Egr-1 open reading frame into plasmid pcDNA3.1/NEO expression vector (Invitrogen), was provided by Dr Thomas E. Eling (Laboratory of Molecular Carcinogenesis, National Institute of Environmental Health Sciences, USA). The vectors pcDNA3.1 and pcDNA3.1-Egr-1 were transfected into MCF-7 cells using jetPEI (Polyplus transfection) according to manufacturer’s protocol. Egr-1 shRNA target sequences were designed and verified as specific for Egr-1 by Blast search against the human genome and real-time PCR, respectively (Table I). The vectors pSUPER-control shRNA and pSUPER-Egr-1 shRNA were transfected using jetPEI and stable cell lines were selected using 1–2 mg/ml G418. Several stable clones were isolated after shRNA transfection and individually characterized.

### Statistical analysis

Data were analyzed by the Student’s t-test and P<0.05 was considered statistically significant.

## Results and Discussion

### Induction of Egr-1 by metabolic stress and ROS

We analyzed the gene expression profiling of A549 cells that were treated with GD or GD+PMA by cDNA microarrays (21). One of GD-induced genes was Egr-1 (Fig. 1A); Egr-1 level was increased 3.4-fold during necrosis, whereas its level was not significantly changed during apoptosis. The induction of Egr-1 by GD was also observed in MDA-MB-231 and HepG2 cells that underwent necrosis upon GD, as revealed by RT-PCR (Fig. 1B). We further examined GD induction of Egr-1 in other cancer cells. Western blot analysis showed the induction of Egr-1 by GD in MDA-MB-231 and HepG2 cells, but not in MCF-7 cells that exhibit necrosis to a much lower degree than MDA-MB-231 and HepG2 cells upon GD and in HCT116 and HeLa cells that exhibit apoptosis upon exposure to GD (Fig. 1C). Real-time PCR confirmed the induction of Egr-1 by GD in MDA-MB-231 and HepG2 cells (3- to 4-fold), and but not in MCF-7, HCT116, and HeLa cells (Fig. 1D). GD is known to induce necrosis by increasing mitochondrial ROS production. Thus, we examined the possible role(s) of ROS in GD-induced Egr-1 expression. Egr-1 induction by GD was inhibited by treatment with the antioxidant N-acetylcysteine (NAC) in MDA-MB-231 and HepG2 cells (Fig. 1D). In addition, H_2_O_2_ and menadione (an O_2_^-^ generator) increased Egr-1 mRNA expression in MCF-7 cells as determined by real-time PCR (Fig. 1E), indicating the redox-sensitivity of Egr-1 expression. H_2_O_2_ at non-toxic doses has been shown to induce the accumulation of mRNA for Egr-1 gene in mammalian cells (24).

### Egr-1 shRNA prevented metabolic stress-induced necrosis and HMGB1 release

To explore the role(s) of Egr-1 in necrosis, we examined the effects of Egr-1 shRNA, directed to the C-terminal region of human Egr-1 mRNA sequences (position from 1630 to 1648 in human cDNA, Table I), on GD-induced necrosis. HO/PI double staining method was used to identify apoptosis as well as necrosis. While HO penetrates non-selectively plasma membrane of both damaged and intact cells and binds to DNA, causing a blue nuclear fluorescence, PI penetrates only cells with damaged-membranes, causing red nuclear fluorescence. Thus, the cell death mode could be discriminated morphologically by nuclear fluorescence images: intact blue nuclei, condensed/fragmented blue nuclei, condensed/fragmented pink nuclei, and intact pink nuclei indicated viable, early apoptotic, late apoptotic (secondary necrotic), and necrotic cells, respectively. Egr-1 shRNA appeared to effectively knock down Egr-1 mRNA levels in MDA-MB-231 cells, as determined by RT-PCR (Fig. 2A). Egr-1 shRNA significantly inhibited GD-induced cell rounding (data not shown) and increase in cell population that had intact pink nuclei in HO/PI staining in MDA-MB-231 cells (Fig. 2B), without increasing the population of the cells with condensed/fragmented blue nuclei and apoptotic bodies (data not shown). Thus, knockdown of Egr-1 appeared to inhibit GD-induced necrosis without switching to apoptotic cell death as an alternative death mechanism. We also observed that Egr-1 shRNA suppressed GD-induced release of HMGB1 into the extracellular space (Fig. 2C). Previously, we showed that in contrast to a general concept that necrotic cell death causes the release of most cellular proteins due to cell membrane rupture, only a restricted set of cellular proteins such as HMGB1 and CuZnSOD were selectively released during GD-induced necrosis (25). Egr-1 shRNA appeared to suppress GD-induced release of CuZnSOD into the extracellular space (Fig. 2C). These results indicate that Egr-1 may be involved in metabolic stress-induced necrosis.

Mitochondrial O_2_^-^ is induced upon GD and mediates GD-induced necrosis and cytotoxicity (26–28). As shown in Fig. 2D, GD significantly enhanced the production of mitochondrial ROS, O_2_^-^, and intracellular H_2_O_2_, as revealed by staining with three different fluorogenic probes including MitoTracker Red CM-H_2_XRos, HE, and DCFH-DA, respectively. Egr-1 interference blocked GD-induced production of mitochondrial ROS, O_2_^-^, and intracellular H_2_O_2_ (Fig. 2D), indicating that Egr-1 may control necrosis through regulating GD-induced mitochondrial ROS production.

### Egr-1 overexpression facilitates GD-induced necrosis

To further examine the role of Egr-1 in necrosis, we overexpressed Egr-1 in MCF-7 cells. Egr-1 is involved in HGF-induced cell scattering, migration, and invasion via Snail activation (19). Egr-1 overexpression in MCF-7 cells caused the morphological changes including loss of intercellular adhesion and formation of a spindle-like cell shape and pseudopodia, which represent the morphology typical of mesenchymal cells (Fig. 3A and B). However, it did not induce necrosis (data not shown). These results demonstrate that Egr-1 is necessary but not sufficient to trigger necrosis. Necrosis is closely linked to excess ROS production, mitochondrial dysfunction, and decreased ATP production (29,30). Thus, Egr-1 may trigger necrosis if tumour cells are under metabolic stress. Therefore, we examined whether Egr-1 overexpression could facilitate GD-inducible necrosis in MCF-7 cells that exhibit a much lower degree (approximately 2–3%) of necrosis upon GD. In MCF-7 cells, Egr-1 overexpression slightly, but to a statistically significant extent (12–13%), increased necrosis upon GD (Fig. 3C), indicating the necrosis-facilitating activity of Egr-1.

### Egr-1 shRNA prevents metabolic stress-induced necrosis in MTSs and suppresses MTS growth

We examined the effects of Egr-1 shRNA on necrosis using MTSs. MTSs closely resemble poorly vascularized solid tumours, and thus are used for an *in vitro* model of solid tumours. MCF-7 cells formed tightly packed spheroids of a homogeneous size and as the MCF-7 MTSs grow, a proliferation gradient is observed, with proliferating cells at the periphery, cell cycle arrested cells in the inner regions, and necrotizing cells in the core regions (31,32). Continued MTS growth leads to the formation of necrotic core due to microenvironmental stresses including deprivation of oxygen and nutrients. H&E and HO/PI double staining revealed the necrotic core formation at 8–9 days of MTS culture (22,33). Although monolayer-cultured MCF-7 cells exhibit limited levels of necrosis upon GD, they showed prominent necrotic cell death in the core region when cultured as MTSs. An increased expression of Egr-1 was detected with extended MTS culture (Fig. 4A); Egr-1 induction was observed at 7 and 9 day MTSs. To determine the expression of Egr-1 in MTSs, the spheroids were selectively dissociated to yield cells from four discrete regions within the spheroid. Enhanced Egr-1 expression was detected in the innermost F4 fraction (Fig. 4B), indicating that Egr-1 expression is closely related to microenvironmental stresses, such as hypoxia and GD. As shown in Fig. 4C, Egr-1 shRNA prevented MTS growth. We further found that Egr-1 shRNA caused a prominent reduction in the population of cells that had pink nuclei with HO/PI staining at 9 days in MCF-7 MTS culture (Fig. 4D). These findings demonstrate that Egr-1 is involved in GD-induced necrosis and tumour progression.

### Biological relevance of this study

An immediate early gene Egr-1 is implicated in tumour cell biology. While Egr-1 is known to induce apoptosis in tumour cells, it also promotes tumour progression, survival, and angiogenesis (6–13). In this study, we showed that Egr-1 is induced upon GD and is implicated in GD-induced necrosis. Egr-1 appeared to be induced by GD-triggered mitochondrial ROS production and to exert a positive effect on mitochondrial ROS production, in a forward feeding ROS-producing fashion. ROS induced under stressful conditions are known to move from a mitochondrion to neighboring mitochondria to enhance ROS production in a process known as ROS-induced ROS release (RIRR) (34,35). Thus, Egr-1 may be implicated in the mechanisms for RIRR, which is responsible for GD-induced necrosis. How does Egr-1 affect mitochondrial ROS production upon GD? Mitochondrial dysfunction has been shown to be linked to increased ROS production and necrosis induction. For instance, tumour cells with dysregulated mitochondria undergo necrosis in response to a glycolysis inhibitor 2-deoxyglucose or alkylating DNA damage that causes rapid ATP depletion (36). Thus, Egr-1 may regulate genes linked to mitochondrial dysfunction. Previously, we showed that Snail (22) and Dlx-2 (37) are also implicated in GD-induced necrosis; thus, Snail, Dlx-2 and Egr-1 may cooperate to induce necrosis. We further showed that Snail suppressed mitochondrial respiration and cytochrome C oxidase (COX) activity by inhibiting the expression of 3 COX subunits, including COXVIc, COXVIIa, and COXVIIc (38). Because Egr-1 is able to induce Snail (data not shown), Snail may be responsible for Egr-1-triggered necrosis. The mechanism whereby Egr-1 and Snail enhance mitochondrial depression, mitochondrial ROS production, and necrosis is under investigation.

## Figures and Tables

**Figure 1:** Induction of Egr-1 during GD-induced necrosis. (A) A549 cells were pretreated with PMA and treated with GD for 12 h and microarray analysis was performed. The numbers mean fold increase in expression as compared with GD-untreated control cells. (B) MDA-MB-231 and HepG2 cells were exposed to GD medium for the indicated times, and then analyzed by RT-PCR for Egr-1 and GAPDH. (C) Several cancer cells including MDA-MB-231, HepG2, MCF-7, HCT116, and HeLa were exposed to GD for the indicated times, and then analyzed by western blotting for Egr-1 and α-tubulin. (D) Cancer cells were pretreated with NAC (10 mM) for 1 h, exposed to GD medium for 12 h, and then analyzed by real-time PCR for Egr-1 and β-actin. Results are expressed as mean ± SE. ^**^P<0.01 versus untreated; ^##^P<0.01 versus GD-treated cells. (E) MCF-7 cells were treated with H_2_O_2_ (300 μM) or menadione (O_2_^-^, 10 μM) for the indicated times and then analyzed by real-time PCR for Egr-1 and β-actin. Results are expressed as mean ± SE. ^*^P<0.05, ^**^P<0.01 versus untreated.

**Figure 2:** Egr-1 plays a role(s) in GD-induced necrosis. (A) MDA-MB-231 cells were stably transfected with control or Egr-1 shRNA and exposed to GD for 12 h and then analyzed by RT-PCR using primers for Egr-1. (B) MDA-MB-231 cells stably transfected with control or Egr-1 shRNA were exposed to GD for the indicated times, and stained with HO/PI, and observed by fluorescence microscopy, and apoptotic and necrotic cells were scored. Results are expressed as mean ± SE from 500 to 800 cells per treatment group and from three independent experiments. ^**^P<0.01 versus control; ^#^P<0.05, ^##^P<0.01 versus control shRNA. (C) MDA-MB-231 cells stably transfected with control or Egr-1 shRNA were exposed to GD for 12 h and the media were analyzed by western blotting with antibodies against HMGB1, CuZnSOD, ERK, and α-tubulin. (D) MDA-MB-231 cells stably transfected with control or Egr-1 shRNA were exposed to GD for 3 or 6 h, and mitochondrial ROS and O_2_^-^ and intracellular H_2_O_2_ production was measured using the MitoTracker Red CM-H_2_XRos, DHE, and DCFH-DA, respectively, under a fluorescent microscope (X200, Carl Zeiss). Results are expressed as mean ± SE. ^*^P<0.05, ^**^P<0.01 versus untreated; ^#^P<0.05, ^##^P<0.01 versus control shRNA.

**Figure 3:** Egr-1 overexpression triggers GD-induced necrosis in MCF-7. (A and B) MCF-7 cells were transiently transfected with a pcDNA3.1-Egr-1 expression vector for 48 h and Egr-1 expression was analyzed using RT-PCR and real-time PCR (n=3) for Egr-1 (A) and the cell morphology was examined using phase-contrast microscopy and photographed under magnification ×100–400 (B). (C) MCF-7 cells transiently transfected with pcDNA3.1-Egr-1 plasmid for 5 days were exposed to GD for 12 and 18 h and then stained with HO/PI and observed under a fluorescence microscope and apoptotic and necrotic cells were scored. Results are expressed as mean ± SE from 500 to 800 cells per treatment group and from three independent experiments. Results are expressed as mean ± SE. ^**^P<0.01 versus Mock.

**Figure 4:** Egr-1 shRNA inhibits the growth of multicellular tumour spheroids (MTSs). (A) MCF-7 spheroids were seeded into 1.2% agarose-coated 96-well plates at a density of 400 cells per well and cultured for up to 9 days. The MTS was analyzed by real-time PCR for Egr-1 expression. The values are expressed as mean ± SE (n=3). ^*^P<0.05, ^**^P<0.01 versus two-dimensional cultured cells. (B) After 7 days of MCF-7 MTS culture, the MTSs were dissociated into subpopulations of cells from different locations in the spheroids, as described in Materials and methods. The isolated cells were analyzed by RT-PCR using primers for Egr-1 and GAPDH. (C) MTS of MCF-7 cells stably transfected with control or Egr-1 shRNA were cultured for up to 9 days. To calculate MTS size, diameters of five spheroids were measured every day. Results are expressed as mean ± SE. ^**^P<0.01 versus control shRNA. (D) MTS of MCF-7 cells stably transfected with control or Egr-1 shRNA were cultured for 7 and 9 days and the cells were isolated and stained with HO/PI and apoptotic and necrotic cells were scored. Results are expressed as mean ± SE from 500 to 800 cells per treatment group and from three independent experiments. Results are expressed as mean ± SE. ^**^P<0.01 versus 7 days MTS; ^**^P<0.01 versus control shRNA.

**Table I:** Sequences used in this study for RT-PCR, real-time PCR, and shRNA interference.

		Sequence 5′→3′	Annealing temperature (°C)
RT-PCR			
GAPDH			
NM_002046.3	Sense	GTGGTCTCCTCTGACTTCAAC	
	Antisense	TCTCTTCCTCTTGTGCTCTTG	
Egr-1			
NM_001964.2	Sense	ATTCTGAGGCCTCGCAAGTA	54
	Antisense	CACTGCTTTTCCGCTCTTTC	
Real-time PCR			
β-actin			
NM_001101.3	Sense	ACTCTTCCAGCCTTCCTTCC	
	Antisense	TGTTGGCGTACAGGTCTTTG	
Egr-1	Sense	AGGACAGGAGGAGGAGATGG	62
	Antisense	GGAAGTGGGCAGAAAGGATTG	
shRNA interference			
Con shRNA		AATTCTCCGAACGTGTCACGT	
Egr-1 shRNA		AAGTTACTACCTCTTATCCAT	
